# Disaster risk management system in Vietnam: progress and challenges

**DOI:** 10.1016/j.heliyon.2022.e10701

**Published:** 2022-09-25

**Authors:** Tran Thi Lan Huong, Duong Thi Van Anh, Tran Tho Dat, Dinh Duc Truong, Duong Duc Tam

**Affiliations:** a The National Economics University (NEU), Hanoi, Viet Nam; b France Vietnamese Centre For Management Education (CFVG), NEU, Viet Nam

**Keywords:** Disaster risk management, Climate change, Disaster prevention, Flood, Storm, Drought, Institution arrangement

## Abstract

**Background:**

Vietnam is one of the countries most impacted by disasters in Asia- Pacific. Floods, droughts and storms are the most common catastrophes. These risks endanger millions of lives and create massive financial and production losses.

**Objective:**

This study aims at reviewing the disaster risk management (DRM) system in Vietnam, identifying progress and challenges of this system, hence making recommendations for improving the system for better responding with natural hazards.

**Method:**

The study uses PSR model (Pressure- State- Response) in combination with DRM management framework by United Nations Development Program (UNDP) to evaluate DRM system in Vietnam with 5 aspects: (i) DRM regulatory framework (ii) DRM organization (iii) DRM financial resources (iv) DRM integration in to plans at central and local levels (v) Disaster warning and education. The data collection consists of reviewing existing literature and interviewing key informants in DRM.

**Results:**

Disasters is a serious threat to Vietnam’s socio economic development. To respond, Vietnam has made many efforts including develop a comprehensive legal framework for DRM which Law on Disaster Prevention and Control takes the key role. Vietnam has also established a fairly well organized DRM system from the central to local levels. The financial sources for DRM are arranged from State budget and sources outside State budget. Vietnam has developed major policies for integrating DRM into development plans centrally and locally. The disaster information and warning system is being modernized with the integration of disaster education in training programs. Challenges in DRM are identified, including institutional, financial and information issues. In addition, Vietnam is facing the increase of disasters and extreme climate events due to climate change. Covid 19 and its socio-economic consequences also lead to a lack of resources for DRM. Economic development moreover results in the decline of ecosystem-based disaster mitigation works and put more pressures on DRM.

**Recommendations:**

In the future, Vietnam should develop an information-sharing network between ministries, sectors, localities and NGOs to support the policy formulation process and enhance the coordination of multi-stakeholders. The country should also establish more proper funding allocation mechanisms to fulfill DRM’s demands, especially for disaster preparedness and reconstruction phases.

## 1 Introduction

Vietnam is one of the most disaster impacted countries on the planet [1, 2]. With a long coastline of 3240 km, combining with diverse topography, Vietnam faces with high disaster risks, ranking 91 out of 191 countries by 2019 INFORM Risk Index. The country has extremely high exposure level to floodings, including riverine, flash and coastal flooding. Vietnam also has high exposure to tropical cyclones and their associated hazards. Drought risk is slightly lower but still significant as highlighted by severe droughts during 2017–2021 [3, 4, 5]. In the flood period from October to late December, Central region is the most influenced by flooding [6, 7]. It is reported that nearly 70% of the national population living in coastal provinces and low deltas, making them vulnerable to flooding [8, 9].

The impact of natural disasters to Vietnam is very serious and is an existential threat to national goals of poverty reduction, Millennium Development Goals and sustainable development. Only in the last 10 years, natural disasters have caused significant damage, killing and missing more than 9500 people, and economic losses are estimated at 1.5–1.8% of GDP/year [9, 10].

Recently, the Vietnamese Government has been working hard for disaster risk reduction (DRR) [10, 11, 12]. It has issued several important legal documents, plans and policies to manage disaster risks. Vietnam also collaborates closely with neighboring countries for disaster risk control [13, 14, 15]. The Vietnamese National Strategy for Disaster Prevention, Response, and Mitigation to 2020 is critical in mobilizing social resources for disaster prevention response and mitigation [16, 17].

Currently, innovative management strategies have been used by many countries in various fields from Covid control to human resource and crisis management [18, 19]. These studies show that knowledge sharing and creativity are essential elements in the development of innovative strategies for dealing with social challenges. In addition, multiple interventions and the mixed precautionary measures are useful to achieve a significant impact on sustaining and controlling these. Also, social support is positively and significantly associated with adjustment in social and individual behaviors toward efficient management. These empirical evidences can be valuable lessons that Vietnam can apply in crisis managing, including DRM.

This paper analyzes the DRM system in Vietnam. With a typically political system, the disaster management model in Vietnam also has its own characteristics. This research is an attempt to address the following questions:

- What is the status and damage caused by natural disasters in Vietnam?
- What are the components of the DRM system in Vietnam, how is it operating and what are its achievements?
- What challenges is Vietnam facing in DRM?
- What strategies and solutions need to be implemented to promote effective DRM in Vietnam.

## 2 Analytical model and materials

In this study, the theoretical framework employed to analyze the DRM system in Vietnam is PSR model (Pressure- State- Response). The PSR framework was firstly developed by Tony Friend for analyzing the interactions between environmental pressures, state of the environment and environmental responses [17]. Since 1970s, Organization for Economic Cooperation and Development (OECD) applied an adaptive version of this model to its works on environmental reports. The usefulness and relevance of PSR model was then re-evaluated during 1990s when OECD initiated environmental indicators for assessing management performance. In that process, OECD nations agreed that PSR framework was a useful and robust model and should be used in studies on environmental data and indicators by OECD [18].

PSR framework for DRM is based on the idea of causality: disaster exerts pressures on the environment and change its quantity and quality (state). Societies respond to these changes through policies and management solutions (response). In the model, pressure reflects the exposure of the natural and social systems to external factors. State reflects the social and economic impacts to economic systems of the region/nation caused by pressures. Response represents measures taken by societies facing such socio-economic issues such as measures to prevent restore and remedy from negative effects of disaster. At present, evaluations based on PSR model has been widely used in several social, economic and environmental fields [18].

In addition, the study also uses the framework of disaster management system (UNDP 2015) [13] to further analyze the DRM system in Vietnam. According to UNDP, a national DRM system is generally composed of five aspects: (1) laws and regulations; (2) institution arrangement including a set of operational agencies or administrations in charge of implementation; (3) financial resource for DRM; (4) information, education, communication and training (IECT) (5) disaster warning system. In fact, countries might pay attention to some of these aspects in selective manners [19, 20].

To discuss the case of Vietnam in detail, we used the above 5-bloc configuration suggested by UNDP with some adaptations including (i) NDM laws and regulation; (ii) DRM management bodies; (iii) financial resource for NDM; (iv) integration of DRM in management plans at national, provincial and sectoral levels and (v) disaster warning and education.

Combining the PSR model and the disaster management system model by UNDP, the study presents the following analysis diagram (Figure 1). The study also conducts a SWOT analysis of the DRM system from primary and secondary data to propose solutions to improve this system in Vietnam in the context of climate change.

**Figure 1:** Analytical model for DRM system in Vietnam.

Data collection process of this study consists of reviewing existing documents, combined with information collected from in-depth interviews with management officers and experts [21, 22, 23].

In the first step, analysis reports and studies from literature on the related issue were studied. These reports come from Web of Science, reports of World Bank (2017), UNDP (2016), Vietnam Government (2020), Ministry of Finance (MOF) (2019), Ministry of Planning and Investment (MPI) (2019) and ADB (2020) [16, 24, 25].

Second, the author conducted 10 in-depth interviews with DRM stakeholders including managers from the Ministry of Natural Resources and Environment (MONRE), the Ministry of Agriculture and Rural Development (MARD), the General Department of Disaster Prevention and Control, the Ministry of Finance (MOF), MPI, Search and Rescue Committee, National Hydrometeorological Center, Non-government organizations (NGOs) and DRM communication units. The interview contents are related to the actual implementation of DRM policies and solutions, specific challenges in the DRM system and solutions to enhance the effectiveness of DRM in Vietnam.

## 3 Disaster profile and impacts in Vietnam

Geographic location and geographical conditions provide unique climatic features that result in severe and diverse disasters in Vietnam. Disasters strike the country virtually every year. Each season has its own set of calamities, and each location has its own set of personalities. Flood, storm, drought, whirlwind, flash flood, coastal erosion and landslide are most common catastrophes (Table 1) [17, 26, 27].

**Table 1:** The level of natural disasters in regions in Vietnam.

	Coastal Economic Zone	Red River Delta	Northeast and Northwest	North East South	Central highlands	Mekong River Delta	South Central Coast
Flood	++++	++++	-	+++	+++	+++++	+++
Storm	++++	++++	+++	+++	++	+++	++++
Whirlwind	++	++	++	++	+	++	++
Drought	+++	+	+++	+++	++	+	+++
Saline intrusion	++	+	-	++	+	+++	++
Inundation	+++	+++	-	++	-	+++	++
Storm surge	++	++	-	++	++	+++	++
Flashflood	+++	-	+++	+++	+++	+	+++
Landslide	++	++	++	++	+	+++	++

Vietnam is vulnerable to multiple natural hazards. However, flood is the most frequent and deadliest hazard (Figure 2). Water resource in Vietnam expands throughout the country, comprising more than 2,000 rivers and streams, deltas, and basins, running along the Central Coastal areas and Mekong River delta, leading to high exposure level of flooding. From 1990 to 2019, floods were responsible for 70% of all natural disaster related fatalities. Flash floods and water-induced landslides are a hazard in mountainous areas due to greater precipitation rates and variable soil conditions [5, 28, 29].

**Figure 2:** Spatial patterns of flood risk assessment by provinces in Vietnam. Source: UNDP 2015 [13].

During typhoon period, from August to November in central coastal areas, April to September in the southwest region, and September to February in the northern part, Vietnam experiences eight to ten typhoons annually. Typhoons are normally accompanied by tidal waves, high winds, storm surges and wreak disaster damages throughout the country. They also have a significant variability in geographical regions, with coastal and central areas are more vulnerable [12, 31, 32].

Drought is another threat affecting the whole country. Drought in the Central provinces is typically resulted from the lack of rainfall and poor water retention capacity of local reservoirs, exacerbated by sunny and hot weather. Like risks of storms, drought tends to impact specific regions of the country depending on regional weather and topography In 2016, Vietnam faced the worst drought in 100 years, partly caused by the El Nino phenomenon. In the 20 worst impacted provinces, about 2 million people received reliefs, including 500,000 residents in the Central Coastal provinces [10, 13].

### 3.1 Economic impacts

Natural disasters can deceases economic development and affect the ability of countries to maintain positive trends due to wide range of impacts that disasters pose on natural and socio-economic systems [30, 40, 41]. Vietnam is ranked highly in the Asia Pacific region for its relatively rapid growth economy for the last 30 years. However, the country has been suffering significant disasters affecting macroeconomic variables, public finance conditions and longer-run fiscal health [3, 17]. Over the period 1989–2019, Vietnam experienced an average annual losses of 1.2–1.5% of total GDP (Figure 3). Overall, storms floods and have resulted in the largest economic damages with their impacts [1, 31].

**Figure 3:** Economic loss caused by disasters and its cost per GDP. Source: UNDP (2015) [5].

Catastrophes may also impose long-run obligations of the Vietnamese government public finance, affecting total spending and fiscal balances. In spite of current provisions of budget at national and provincial levels setting aside 2–4% of available funding resources for disaster prevention and preparations, the expenses of recovery and restoration often exceed financing capacity [13].

### 3.2 Social impacts

Vietnam vulnerability to disasters is enhanced by the country levels of poverty. ADB (2013) highlighted that many households have high probability of falling into extreme poverty even when they expose to fairly high frequency of hazards. A disaster at frequency of once in five years can push 30% household into extreme poverty. While many families have not the same exposure levels, disasters threaten to increase exposure through their impacts with extreme events.

World Bank (2018) suggested that floodings in urban areas affected most strongly the poorest communities due to these areas are high hazard exposure while having low levels of adaptive capacity. In addition, gender is also connected to this issue. Women tend to be most vulnerable to the risks since living in precarious environment [42]. Similar problems are identified in flood-prone rural areas, especially in Red and Mekong deltas where the poor and landless families have lowest resilience. The communities with most sensitivity to disaster impacts also include ethnic minority groups who are facing more challenges to their adapting capacity. Poor communes are usually the most dependent on nature and ecosystems to maintain their livelihoods. Those functions can be destroyed by disasters, and also be determined partly by adaptive measures.

The impact of disasters is also of particular concern in urban areas – where the population is densely populated and is socio-economic development center of the province, region and the whole country. Over the last 20 years, the number of cities increased rapidly from 629 cities (1999) to 850 cities (2021) with a current urbanization rate of 41.5%. If there is no effective response to the high concentration of population, housing, welfare works and infrastructure, the level of vulnerability will increase much. All 5 big cities directly under the central government (Ho Chi Minh, Hanoi, Hai Phong, Da Nang, Can Tho) and coastal areas are strongly affected by disasters. In Ho Chi Minh City, flooding has affected 47% of the poor population. Near to half of the wards and communes are regularly flooded affecting 22% of the city’s population city [18, 20].

Different parts of population suffer disproportionate and different disasters' social impacts. In Vietnam, catastrophe impacts vary although the nation is made up with heterogeneous people groups from many social contexts, with different levels of access to support, services and capitals. Disparities between urban and rural regions are still obvious, affecting access to services, public facilities; availability of support and adaptive capacity to extreme disasters, as well as local households' assistance in dealing with chronical stresses from accumulated and prolonged impacts. In addition, the poverty situation is also varied across geographical regions; with high rate of the poor in the northern mountainous provinces and rural communes (see Figure 4).

**Figure 4:** Poverty rate by provinces in Vietnam. Source: UNDP (2015) [15].

However, poverty situation is not the only variable affecting the severity of hazard impacts in the country. One research about the relationship between of welfare of households and disasters showed social factors related to hazard impacts depend on population groups and demographics. E.g. it is fairly obvious that the damages of disasters to the Kinh families, (dominated ethnic group in Vietnam) are significantly lower than those of other ethnic minorities' households. Education is also a factor significantly determining the degree of resilience to disasters, higher education households are more resilience against droughts and floods than low education families due to better ability to prevent, prepare and recover from disaster impacts [13, 15].

Industrialization and rapid urbanization process also increases pressures on the resilience of urban system in some regions. Migration to urban areas and cities for employment opportunities has contributed to quick expansion of cities, while local governments often do not have sufficient capacities to satisfy increasing needs of city services and housing. Uncontrolled settlement areas generate slums in cities represent the deteriorated conditions of the poor in urban areas. They are the most vulnerable groups to disasters and environmental pollution. Effects of recent floods might cause contingency damages in healthcare sector, particularly after big disasters. Moreover, lacking of access to clean water usually spreads of vector-borne diseases (e.g. cholera, diarrhea, typhoid etc. [21, 23]).

## 4 Natural disaster risk management system in Vietnam

### 4.1 Regulatory framework for DRM

Vietnam has made many efforts to develop a legal document system on DRM and extreme climate phenomena. In 2007, Vietnam issued the National Strategy for Natural Disaster Prevention and Mitigation until 2020. In 2008, the Government approved the National Target Program on Climate Change (NTPCC) under Decision No. 158/2008/QD-TTG [32]. 2013 marked a turning point in DRM work in Vietnam when the National Assembly passed the Law on Natural Disaster Prevention and Control (LDPC). This Law, coming into effect in 2014, is the first Law on DRM in Vietnam and provides the core principles and components of the nation’s DRM system. As regulated in the Law, DRM activity consists of prevention, response and remediation of disasters' damages and consequences. The Law also assigns roles and responsibilities among ministries, local authorities, domestic stakeholders and other key actors in DRM, especially in disaster prevention and response.

In recent years, the Government has launched many important law papers, policies, and programs to address disaster risk reduction (DRR) and climate change adaptation (CCA) (Table 2). The LDPC, the National Strategy for Natural Disaster Prevention, Response, and Mitigation to 2020, and the NTP-RCC are the most important legal documents in disaster prevention, restoration and control in climate change context. They mention detail issues relating to DRM and promote the integration of DRM contents into plans at national, sectoral and provincial levels [5, 17].

**Table 2:** Some important legal document for DRM and climate change management.

Issue time	Document name	Decision	Effective time
2004	Strategic Orientation for Sustainable Development (Vietnam Agenda 21)	Decision No. 153/2004/QD-TTG	From 2004 onwards
2006	National Water Resources Strategy Towards the Year 2020	Decision No. 81/2006/QD-TTG	2006–2020
2008	National Target Program (NTP-RCC) to respond to climate change	Decision No. 158/2008/QD-TTg	From 2009 onwards
2011	National strategy on climate change	Decision No. 2139/QD-TTG	2012–2050
2012	National Target Program to Respond to Climate Change 2012–2015 Period	Decision No. 1183/QD-TTG	2012–2015
2012	National Action Plan on Climate Change for the period 2012 to 2020	Decision No. 1474/QD-TTG	2012–2020
2012	Sustainable Development Strategy of Vietnam for the Period 2011–2020	Decision No. 432/QD-TTG	2011–2020
2012	National strategy on green growth for the period 2011– 2020 with a vision to 2050	Decision No. 1393/QD-TTG	2011–2020 and vision to 2050
2012	National Strategy on Environment Protection to 2020, with visions to 2030	Decision No. 1216/QD-TTG	2012–2020 and vision to 2050
2012	Management of GHG emissions; management of carbon credit trading activities to the world market	Decision No. 1775/QD-TTg	2012–2020
2013	Resolution on the active response to climate change and the improvement of natural resource management and environmental protection	Resolution No. 24-NQ/TW	2013–2020
2014	Plan for the implementation of national environmental protection strategy by 2020, with a vision to 2030	Decision No. 166/QD-TTG	2014–2020 and vision to 2030
2014	National Action Plan on Green Growth in Vietnam for the period of 2014–2020	Decision No. 403/QD-TTg	2014–2020
2016	Plan for Implementation of the Paris Agreement	Decision No. 2053/QD-TTg	2016–2030
2017	National Action Plan to implement the 2030 Agenda for SDGs	Decision No. 622/QD-TTg	2017–2030
2017	National Target Program for Climate Change Response and Green Growth for the 2016–2020 period	Decision No. 1670/QD-TTG	2016–2020

### 4.2 Institutions and organizations for DRM in Vietnam

DRM requires the participation of many levels, sectors from central to local, domestic and international civil society organizations. According to UNDP in 2015 [13], Vietnam has set up a good DRM organization system from the central to local levels, constantly strengthened to face with the increasing disaster challenges. The organizations of this system have obvious tasks and operational regulations in coordination and administration. The hierarchical institutional structure in DRM includes four levels (national, provincial, district and commune levels), shown in Figure 5.

**Figure 5:** Organizational system for DRM in Vietnam.

At central level, the Central Steering Committee for Natural Disaster Prevention and Control (CCLDPC) is the main policy and decision-making body led by Vietnam Disaster Management Authority. Besides CCLDPC, National Committee for Incident, Disaster Response, Search and Rescue (VINASARCOM) is the Government’s focal Agency for search and rescue, responsible for assisting the Prime Minister in coordinating ministries, sectors, and provinces in their work of disaster search and rescue. The Committee is under the Office of the Government, Chairman of the Committee is the Deputy Prime Minister. The Committee also has other vice-chairmen, including the Ministry of Transport, Ministry of Public Security and MARD. Members include 10 Ministries and Voice of Vietnam, Television of Vietnam and Vietnam Women’s Union. When disasters occurring, VINASARCOM and CCLDPC coordinate to organize rescue actions. In Ministries, 2 above agencies merge into the Department of Flood and Storm Control and Search and Rescue, cooperating and coordinating with VINASARCOM and their provincial offices [26, 27].

### 4.3 Finance for DRM in Vietnam

The financial sources for DRM in Vietnam include 2 main sources including (i) financial sources from State budget, (ii) financial sources outside the State budget.

### 4.4 Financial sources from state budget

#### 4.4.1 State budget contingency

National and local budget contingency are the main source for DRM in Vietnam. Since 2017 (when State Budget Law took effect), the budget contingency is regulated from 2% to 4% of the total annual budget at all administrative levels. The State budget contingency is spent for “preventing, combat and overcoming consequences of disasters, epidemics, hunger relief; important national defense and security and other necessary tasks” [16].

From 2014 to 2019, the total contingency budget for DRM was from 1.91% to 2.39% of the total State budget spending (highest in 2014). These percentages are in line with the regulation of State Budget Law. Although the total volume of contingency budget is quite big, it is normally used for different social purposes and not only for hazard prevention and damage restoration. These details of contingency budgets in Vietnam are shown in Table 3.

**Table 3:** Contingency budgets for disaster management during 2014–2019 (trillion VND).

Year	Estimated State budget contingency			Estimated total state budget expenditure	% of contingency against total state budget expenditure		
	Total	Central level	Provincial level		Total	Central level	Provincial level
2014	23,400	10,800	12,600	978,000	2.39	1.10	1.29
2015	19,200	10,300	8,900	1,006,700	1.91	1.02	0.88
2016	25,000	13,000	12,000	1,147,100	2.18	1.13	1.05
2017	26,000	12,500	13,500	1,273,200	2.04	0.98	1.06
2018	29,300	15,800	13,500	1,390,480	2.11	1.14	0.97
2019	32,097	15,800	16,297	1,523,200	2.11	1.04	1.07

### 4.5 Financial Reserve Fund (FRF)

In the cases that the central government and localities have already spent all of the budget reserve but still are not enough to deal with the consequences of a natural disaster, the central government and the provinces may use FRF to meet expenditure needs of natural disasters. repair and recovery. However, the maximum spending level in the year cannot exceed 70% of the fund’s opening balance at the beginning of the year. As the rules, the balance of the Financial Reserve Fund at each level cannot exceed 25% of the annual budget expenditure estimate of that level. However, at present, the FRF has a rather limited size due to budget overspending for many years. According to MOF (2020), total amount of FRF is only accounted for 0.04% of the total spending budget in period 2010–2019 [33, 34].

### 4.6 National reserve (NR)

NR is State strategic reserve in order to meet proactively urgent demands on prevention, combat and restoration of disasters and epidemics' damages and consequences. The NR system is set at the central level and strategic areas to meet quickly financial requirements in urgent situations, managed by MOF. The fund for NR is collected from State budget determined by Vietnamese Assembly.

NR Strategy to 2020 strengthens the NR potential to guarantee that by 2020 it will reach about 1.5% of GDP. So far, the total NR is about VND 15,000 billion, increasing nearly 1.5 times in comparison with 2010. However, the size of NR tends to fall. Total value of NR in 2019 reached nearly 0.2% of total GDP, very low compared to the set Strategy target. So, with this NR fund, it is challenged for Vietnam to respond proactively to urgent demands for disaster recovery, especially when unexpected large-scale situations occur [35].

### 4.7 Sources outside state budget for DRM

#### 4.7.1 Fund for Natural Disaster Prevention and control (FLDPC)

According to the Decree 94/2014 by Vietnamese government, FLDPC is a fund established at the provincial level and managed by the People’s Committee of the province. The fund does not include and originate from the state budget. The money of FLDPC includes:

• Economic units with independent system of accounting: The mandatory contribution amount for a year is 2/10,000 of the total asset value of the units, and must be at least VND 500,000 VND or maximum VND 100 million.
• Citizens from 18 to 65 years: (i) Public and private employees pay 1 day salary/head/year; (ii) Other kind of staffs have to pay 15,000 VND/head/year.

Currently, this fund is employed to support hazard prevention and restoration actions with priorities: (i) support emergency reliefs in drinking water, food, medicine; (ii) support the restoration of health care facilities, houses, schools; (iii) support the sanitary treatments in impacted areas.

#### 4.7.2 Financial support from abroad

Vietnam so far has been receiving very good supports from international organizations and donors in dealing with consequences and damages of disasters. Supports are made in funds and in-kind contribution such as drinking water, food and medicine. Since this is the support outside national budget, so data are not so completed and consistent. Since 2000s, USAID has been providing more than $20 million for DRM assistance and emergency relief and in Vietnam.

Moreover, other international institutions such as the ADB and World Bank have given loans to support the restoration of major infrastructures damaged by hazards. In 2015, ADB provided Vietnam with a fund of USD 20 million for infrastructure improvement, and this fund was subsequently used to assist provinces seriously damaged by disasters. In 2017, the World Bank gave a loan of USD 358 million to Vietnam for implementing the project Emergency Post-Disaster Reconstruction to help restore infrastructures in Quang Nam, Binh Dinh, Quang Ngai, Hue and Ha Tinh provinces. These are the provinces suffered heavy damages from prolonged floodings in 2016. The project helps to restore and rehabilitate roads, bridges, irrigation systems, water supply systems and disaster prevention works. The project helps improving the capacity of DRM, benefits 1.2 million residents in 5 above provinces.

### 4.8 Integrating DRM into plans and policies in Vietnam

From early 2000s, when disasters became more frequent and severe, Vietnam had critical guidelines and policies for integrating DRM into the National Socio-economic Development Plan (SEDP). In addition, LDPC also stipulates the integration of DRM into sectoral and provincial SEDP (Articles 4). The NTP-RCC sets out to integrate natural disaster and climate change into strategies, master plans, programs and SEDP [13, 38]. In addition, the Law on Dikes (2006), Law on Environmental Protection (2013), Law on Water Resources (2012), Law on Forest Protection and Development (2004), Law on Land (2013), Law on Mineral Resources (2010), Law on Fisheries (2003), Ordinance on Exploitation and Protection of Irrigation Works (2001) all mention the integration of DRM into the national, sectoral and local SEDP [13, 17].

Over the years, many Ministries and sectors have pioneered the compilation of guidelines for integrating DRM into the sector’s development policy and planning. For example, in 2012, MONRE presided over the compilation of Technical Guidelines for mainstreaming climate change into developing development strategies, plans, and master plans. In 2013, MPI compiled a Guide to Prioritizing Climate Change Adaptation Investment (APRT) in the SEDP process. The MARD has formulated the Sector Development Plan for 2010–2020 based on logical framework design, associated with national and ministerial-level programs to implement comprehensively, with focus and focus. In 2011, the “Action plan to respond to disasters and climate change of the Agriculture and Rural Development Sector for 2010–2020 with a vision to 2050” was issued.

For the construction and industry sectors, the industry’s main tasks and solutions directly related to DRM are the formulation and implementation of construction and industry planning, especially in areas frequently impacted by disasters. However, so far only 43 provinces and cities have made urban and rural planning. Besides those integrated guidelines and policies, localities and sectors have organized many seminars, training courses and communication to strengthen capacity on DRM.

In addition to integrated guidelines and policies, sectors and localities have organized many training courses, seminars and communication activities to strengthen their capacity on DRM. Currently, localities and sectors have been implementing action plans to implement the National Strategy on Disaster Prevention and Mitigation until 2020 and the Community-Based Disaster Risk Reduction Project [13, 17].

Overall, national long-run DRM vision is currently significantly aligned with Sendai Framework, SDGs and Paris Climate Agreement. Viet Nam has made progresses in including these frameworks in critical regions like Red River and Mekong Delta. Especially, the Government Resolution 120 /NQ-CP on “Sustainable and Climate-Resilient Development of the Mekong Delta” in 2017, represents the commitment of Vietnam towards a sustainable development of Mekong Delta which is based on diversifying and greening economic actions, while increasingly invest in mitigating negative impacts of natural disasters.

### 4.9 Disaster warning and education about DRM

#### 4.9.1 Disaster early warning system

Early warning of natural disasters plays a decisive role in the effectiveness of prevention and reduction of risks caused by disasters to the socio-economic system. Over the years, Vietnam has achieved a number of achievements in building and perfecting this system. Firstly, the hydrometeorological legal system has been gradually improved, creating an important legal corridor, ensuring regular and continuous operations of the whole national hydrometeorological forecasting system, from monitoring, information transmission to forecasting. notice, warning. Since 2016, implementing Circular 41 on regulations and procedures for forecasting and warning of dangerous hydrometeorological phenomena, the number of forecasted types of natural disasters has increased significantly, including: Storms/Twilights, large-scale heavy rains, flood, inundation; flash floods, landslides, land subsidence due to rain, flood or runoff; cold; hot; drought; saline intrusion, thunderstorms, lightning, storms, whirlwinds, hail and local heavy rain; coastal fog, high waves, storm surge, storm surge, monsoon and storm surge. Secondly, the hydrometeorological monitoring network has been upgraded to be modern and synchronous. Gradually switching from manual to automatic measurement, knitting monitoring stations in mountainous and remote areas, has played a role in ensuring timely provision of data for the monitoring of hydrometeorological phenomena. Good service for disaster prevention and control. By 2020, the national monitoring network has 284 surface meteorological stations; 29 agricultural meteorological stations; 14 radiation stations; nearly 2000 automatic rain gauge stations; 359 hydrological stations; 27 hydrometeorological stations; there are 180 environmental measurement stations/points; The network of meteorological stations does not include: 06 radio-air sensing stations, 08 overhead wind measurement stations by optical theodolite, 03 stations measuring total amount of Ozone - Ultraviolet radiation and 10 weather radar stations spread all over the world. all over the country, 18 lightning positioning stations. Thirdly, strengthen early, long-term forecasting. The hydrometeorological sector has extended the time limit for weather forecasting and early warning of natural disasters to 10 days; The content and format of the newsletter has changed a lot, focusing on providing forecast information on a smaller scale (district, commune level) and longer time period [3, 18].

Vietnam has also set up a nationwide Early Warning System (EWS) from central to local levels. At central level, the CCLDPC and VINASARCOM coordinate disaster warning, response and restoration activities. At regional level, Flood and Storm Control Centers in Ho Chi Minh City and Da Nang support MARD Standing Office of the CCLDPC coordinating information flows between central and provincial levels. CCLDPC and VINASARCOM members are set under one combined Provincial Committee for Flood and Storm Control and Search and Rescue at the commune, district and provincial levels. Of which, the MARD has responsibilities for disaster response, while MONRE has responsibilities for disaster forecasting [3, 13, 26].

EWS Innovations in Vietnam has included SMS text messaging. Any people and communities can reach out to government management agencies to register their phone number for free SMS warning information. Through DRM work, many NGOs such as Vietnamese Save the Children have collaborated with local agencies and communication companies to develop EWS text messaging providing weather and disaster information to potentially vulnerable provinces, including Ha Tinh, Thua Thien Hue, Quang Nam, Quang Binh and Da Nang. In the past, coastal communities disseminated disaster information or emergencies through loudspeaker systems in commune public spaces or through commune leaders carrying out household visits. Mobile devices currently have been registered to communicate with district and provincial departments through free SMS. This innovation enables volunteers getting SMS warning immediately and then informing others as needed. They might also transmit data on disasters and other situations in their regions to help improve data collecting, risk mapping and disaster decision-making [36].

#### 4.9.2 Education on DRM

Globally, during the implementation of Hyogo Framework for Action during 2010–2020, nations commit to and progress toward 5 national priorities for actions to the safety of children. In Vietnam, the MARD and the Ministry of Education and Training (MOET) launch a five-year program (2018–2023) to strengthen preparedness ability of schools for natural disasters. The program aims at equipping students and teachers with the knowledge of preparation for disasters. In 2017, Vietnam Disaster Management Authority and UNDP instituted the campaign “Schools of Son Tinh” which equipped about 5000 students in regions vulnerable to storm surges and floods with knowledge and skills for saving their lives [17, 31].

Save the Children (SC) has also complimented this activity to develop risk reduction capacity for children and teachers, linking communities and schools. SC aims at supporting the integration of disaster preparedness into curriculums of schools. It has been working with partners in the MOET and international organizations for producing guidebooks to include DRR into schools' programs. In disaster-prone areas, SC is working specifically for providing children with life-saving swimming skills and introducing floating backpacks to protect pupils in flash flood area.

## 5 Challenges in NDM system in Vietnam

### 5.1 Legal and institutional challenges

According to UNDP [13], the current system of documents on DRM is quite cumbersome. Only regulations related to flood and storm control have more than 150 documents. Still, most of them are sub-law documents, not enough to deal with society’s major and pressing problems related to combating and mitigating the harmful effects of disasters [17].

The LDPC regulates organization, tasks, powers and coordination mechanism of CCLDPC and VNSARCOM with disaster management agencies in ministries and localities, however currently in Vietnam, the coordination among sectors still has many limitations due to “*lack of synchronous planning and cooperation among ministries, branches, and localities*” and “*lack of timely adjustment in policy on mobilizing resources for prevention and mitigation disasters*” [37, 38]. DRM management activities, including prevention, response and remediation of hazard consequences; however, it does not emphasize much on mitigation. Where mitigation can help reducing the disasters' consequences before occurring, the current approach is fairly reactive. A more proactive DRM approach would allow preparedness, mitigation, and early warning for hazards before they occur and might help vulnerable communities become safer and response better to disaster.

In addition, the limitation of human resources, especially at local levels is also recognized as a big challenge in the process of integrating DRM into development plans at subnational levels. Moreover, some areas of DRR and CCA is overlapping, the synergies has not been well-recognized because of aforementioned issues relating to capacity lacking [1]. At central level, inter-ministerial agencies in charge of DRM implementation and planning often lack financial resources and authority. Thus, it is required that the coordination to implement CCA and DMR mandates should be improved at all levels.

### 5.2 Financial challenges

Firstly, Vietnam is facing a huge shortage of financial resources for disaster prevention. The LDPC clearly states that disaster prevention is the focus of priority. However, Vietnam currently has not been spending properly for hazard prevention activities. As a result, the hazard prevention capacity of stakeholders is poor, especially at local levels. The existing finance capacity only fulfills around 20% of the anticipated emergency and recovery demands. This protection gap exist beyond disaster damages, resulting in higher production, property and livelihoods losses.

Secondly, Vietnam does not have enough financial resources to reconstruct after disasters with great damage (extreme phenomena). Hence, it is hard to restore the production and economic capacities of impacted sectors, localities and households. This situation is leading to an amplification of indirect economic damages in the long run. Disaster financing currently focuses on disaster relief and recovery actions (very short period after the occurrence of disasters). Moreover, districts and provinces' DRM funding still heavily dependents on the budget from Central to cover damages and losses in spite of having local contingency budgets. Table 4 presents the lack of finance for reconstruction after disasters for the period 2012–2018. The fund from state budget is not enough for recovery and reconstruction after disasters.

**Table 4:** Estimated financial gap for reconstruction after disasters in period 2012–2018 (billion VND).

Year	2012	2013	2014	2015	2016	2017	2018
Lack of finance for recovery	4570	2180	7112	8058	3249	2686	7789
Finance for reconstruction	6370	3930	8743	10,008	2550	3572	3997
Lack of finance for reconstruction	770	5872	7752	7149	11,354	17,428	3003

Thirdly, the biggest institutional shortcoming for DRM finance is that there is not yet a central unit that can harmoniously coordinate strategies, policies, and priorities in the DRM plans in short, medium and long-run plans between central and local authorities, between sectors and between regions and provinces in the same natural risk areas. This situation causes financial gaps in DRM priorities and action plans underpinning DRM plans [39].

Fourthly, the planning and budgeting cycle for disasters has many shortcomings: (i) There is no indicator and accounting system the classification of State budget spending for DRM; (ii) Lack of a system to monitor, track and allocate financial flows for DRM; (iii) Lack of assessment and reporting of the results of DMR financing which is the foundation for building DRM mid and long-run fiscal plans.

### 5.3 Challenges in disaster data and information system

Currently, knowledge and data of the links between economic development, human activities and hazard risks is still limited in Vietnam. Increasing disaster risk adds to these challenges because the difficult nature for tracking and predicting the risks, especially in regions lacking data and comprehensive monitoring systems.

Thus, one of the challenges that communities and local authorities are facing when implementing DRM solutions is the difficulty of accessing and capturing DRM information systematically. At the moment, the accessibility level of local authorities and people to hazard information is low. The disaster data/information is only published on certain media that only some certain people could access. E.g. middle-income and rich households usually have easier access to disaster information on the internet than the poor people. Therefore, it is also important to enhance the capacity to access to information for communities and households in vulnerable areas.

In addition, the quality of disaster information and data is still low. Along with supports from international organizations, the Vietnamese government has made a lot of investment on hazard data monitoring and analysis system. However, the temporal and spatial granularity of forecasting and monitoring data can only be used at regional level and can hardly be used at community-level for prevention, response and restoration [43, 44].

### 5.4 Other threats for DRM in Vietnam

In the coming time, DRM work in Vietnam will face identified challenges as follows:

Firstly, natural disasters tend to increase in the context of climate change, especially extreme events. Vietnamese MONRE has just announced the 2020 National Climate Change Scenario. Accordingly, annual rainfall tends to increase nationwide, with a common increase of 10–15% in the middle of the century and 10–20% by the end of the century. In addition, climate change has the potential to change the frequency, intensity, and operating rules of extreme climate events. Some expected results such as the number of storms and tropical depressions tend to increase and have a more concentrated distribution at the end of the storm season. The number of days of extreme cold and harmful cold in the northern mountainous provinces, the Northern Delta, and the North Central region have all decreased. The number of hot days and intense heat tends to increase in most of the country, the largest is in the North Central region, the Northern Delta and the South. Regarding drought, by the end of the 21st century, the number of drought months will increase over most of the North Central region, the Central Highlands and a part of the Northern and South Central Plains and tend to decrease over most of the North Central region. Ministry and Central. Also under this scenario, sea level will rise about 55 cm. The spatial distribution of sea level rise in the East Sea shows that the area between the East Sea (including Hoang Sa and Truong Sa archipelagoes) has significantly higher sea level rise than other areas [45, 46].

Second, the Covid 19 epidemic and its socio-economic consequences lead to a lack of public financial resources to spend on other social goals, including DRM. In Vietnam, the Covid-19 epidemic has experienced four outbreaks and has not ended yet. Vietnam, although it is considered as one of the few countries that responds well to the epidemic, the labor market – employment of Vietnam has also been seriously affected. Vietnam’s economic growth rate has decreased from 6.58% in 2019 to 2.18% in 2021. In the first 7 months of 2021, in 19 southern provinces and cities, where 48% of enterprises in the country accounted for, had up to 79,673 businesses withdrew from the market, an increase of 25.5% over the same period in 2020. As of August, 2021, according to quick reports from southern provinces and cities, there were about 2.5 million workers who had to stop working, accounting for 70% of the number of workers who had to stop working in the whole country [47].

In 2021, the state budget spent 56.27 trillion VND on epidemic prevention. In which, the central government spent 25.35 trillion VND to buy vaccines and to spend on epidemic prevention and control; buy back rice for national reserves already issued to support people facing difficulties due to the Covid-19 epidemic and support localities; localities have spent 30.92 trillion VND from local budgets on epidemic prevention and control and supporting people facing difficulties due to the Covid-19 epidemic. Spending on Covid-19 prevention has led to an increase in overspending and a lack of financial resources to invest in other development goals, including DRM activities.

Third, economic development might lead to the decline of ecosystem-based disaster mitigation works in Vietnam. Ecosystems play an important role in disaster prevention and human protection. Vietnam is one of 16 countries with the highest biodiversity in the world. However, the natural ecosystems in Vietnam are in rapid decline. There are many causes for the degradation of ecosystems in Vietnam, including both direct and indirect causes, such as overexploitation of natural resources, illegal logging, illegal trade. wildlife, infrastructure development activities, agricultural expansion, as well as other economic production activities to serve the increasing needs of people. WWF’s report (2021) shows that, currently in Vietnam 21% of mammals, 6.5% of birds, 19% of reptiles, 24% of amphibians, 38% of fish and 2.5% of vascular plant species are threatened. Over the past 20 years, forested areas have been the most affected habitats with more than 10,544 square kilometers of forest land lost, mainly due to conversion to plantations and fruit trees. About 2.8 million hectares of natural forest has also been lost due to conversion to other commercial crop species. Wetlands are also severely degraded as up to 1 million hectares are destroyed and converted to economic purposes. As these ecosystems decline, their disaster prevention function will also be lost. Since then, the impact of natural disasters on society has become more and more serious [48, 49].

Table 5 summarizes the main points of the SWOT analysis of the DRM system in Vietnam.

**Table 5:** SWOT analysis of DRM in Vietnam.

## 6 Conclusions and recommendations

Vietnam is one of the most disaster impacted nations in the West Pacific region. Natural disasters have been causing significant threats to the livelihoods and lives of millions Vietnamese households. Hence, to reduce the negative effect of catastrophes, it is critical to establish comprehensive disaster preparedness and response strategies for upcoming hazard events.

The DRM capacity of Vietnam has been improved in recent years. The national LDPC and the National Strategy on Disaster Prevention, Response and Mitigation to 2020 are good examples of the country’s efforts to enhance DRM. These efforts are undertaken at the national, provincial and communal levels. Vietnam has also made significant progress in developing institution arrangements and proactive DRM policies as well as mainstreaming DRM into national sectoral and local social- economic development priorities.

Despite much progress, Vietnam’s current DRM scheme still faces significant challenges. Major shortcomings the report identifies include incomplete risk information and ineffective enforcement of related regulations. In addition, the Government still faces a funding gap after disasters.

In the coming time, it is imperative for the country to strengthen its institutional capacities and collaborating mechanisms among regions, ministries and sectors; at the same time developing a more proper financial flow to meet the demands of DRM while further enhancing awareness of local communities in prevention and responding to natural disasters. It is also suggested that developing an information-sharing network to enhance the coordination between multi-stakeholders including disaster management agencies, localities, sectors and civil societies to support the DRM planning and policy formulating process.

In addition, improved financial planning will also be critical to establishing a robust system for disaster preparedness and response. Developing of risk sharing mechanisms such as disaster is insurance is important to protect poverties, livelihoods, infrastructure, and lives from hazards' impacts and provide coverages for sustainably protection of education and health care services as well as employment and agricultural supply chains. It is positive that the Government now has access to a wide range of financial options. However, catastrophe risk reduction and post-disaster response and recovery are heavily reliant on state expenditures at all levels. Greater coordination of these tools might assist the Government in better managing catastrophe expenses and ensuring funds are distributed in an effective and timely way.

## Declarations

### Author contribution statement

Tran Thi Lan Huong & Duong Thi Van Anh: Conceived and designed the experiments; Wrote the paper.

Tran Tho Dat & Dinh Duc Truong: Performed the experiments; Wrote the paper.

Duong Duc Tam: Contributed reagents, materials, analysis tools or data; Wrote the paper.

### Funding statement

This work was funded by The National Economics University, Hanoi, Vietnam.

### Data availability statement

Data associated with this study has been deposited at Mendeley Data under the reserved DOI: https://doi.org/10.17632/zd3tn547hc.1.

### Declaration of interest’s statement

The authors declare no conflict of interest.

### Additional information

No additional information is available for this paper.
